# Educational Psychology Analysis Method for Extracting Students' Facial Information Based on Image Big Data

This article has been retracted.

**DOI:** 10.1155/2022/8709591

**Published:** 2022-05-11

**Authors:** Maoyue Zhang

**Affiliations:** School of Law, Tianjin Normal University, Tianjin 300387, China

## Abstract

At present, most of the research on academic emotions focuses on the concept, current situation, and relevance. There are not many researches on the application of artificial intelligence-based neural network facial expression recognition technology in practical teaching. With reference to image-based big data, this research integrates the application of artificial intelligence facial expression recognition technology with the research on educational theory and applies information technology to the actual teaching process, in order to promote the optimization of the teaching process and improve the learning effect. *Method*. A Hadoop cluster consisting of 3 nodes is built on the Linux system, and the environment required for Opencv execution is compiled for each node, which provides support for subsequent parallel optimization, feature extraction, feature fusion, and recognition of student facial images. The image data type and input and output format based on MapReduce framework are designed, and the image data is optimized by means of serialized files. The color features, texture features, and Sift features of students' facial images and common distractors were analyzed. A parallel extraction framework of student facial image features is designed, and based on this, the student facial image feature extraction under Hadoop platform is implemented. This paper proposes a dynamic sequential facial expression recognition method that combines shallow and deep features with an attention mechanism. The relative position of facial landmarks and local area texture features based on FACS represent shallow-level features. At the same time, the structure of ALexNet is improved to extract the deep features of sequence images to express high-level semantic features. The effectiveness of the facial expression recognition system is improved by introducing three attention mechanisms: self-attention, weight-attention, and convolutional attention. *Results/Discussion*. Through the analysis of the teaching effect, we found that when teachers can obtain the correct student's academic mood, they can intervene on the students' positive academic mood. The purpose of the intervention is to improve the positive academic emotions of students. After the students receive the intervention, their academic emotions are also improved and are positively correlated with their academic performance. Through the analysis of teaching effect, the research can achieve the predetermined goal. From the specific teaching effect of this study, it is concluded that in classroom teaching, teachers should devote energy to intervene in students' positive academic emotions, in order to improve students' positive academic emotions, which will improve students' academic performance and teaching.

## 1. Introduction

The change of the learning environment is often caused by technological innovation first, or the change of the learning environment is ultimately realized through technological innovation [1]. The key technical features of the smart learning environment are mainly reflected in the recording process, situational perception, adaptive interaction, etc., emphasizing the perception and recording of learners' knowledge acquisition and other aspects through motion capture, emotional computing, eye tracking, etc., in order to facilitate learning. Compared with ordinary digital learning environments, smart learning environments focus on cultivating learners' innovative ability, problem-solving ability, decision-making ability, and critical thinking ability, while cognitive activities play an important role in cultivating learners' higher-order thinking ability [2, 3].

In the process of intelligent learning, the emotional state of the learner has an important influence on the learning effect [4]. In addition, the smart learning environment breaks the traditional teaching mode, emphasizing the learner-centered, ubiquitous learning, cloud learning, and seamless learning with MOOC, microcourse, mobile courseware, and electronic teaching materials as learning resources. Learners mostly use intelligent learning terminals such as tablet computers, smart phones, and e-book bags to conduct independent learning or collaborative learning, and teachers and students are mostly in a quasi-separated state in time and space [5]. In traditional teaching, teachers and students have face-to-face and intuitive communication. Teachers' satisfied expressions, words of praise, and gestures of encouragement can convey positive emotions to learners, so as to affect learners' interest and attitude in learning [6]. Due to the quasi-spatiotemporal separation between teachers and students in a smart learning environment, it will be difficult for teachers and students to feel each other's emotions and states, and there is a common problem of “emotional lack” [7]. If the intelligent learning environment cannot organically combine the two, the effective progress of intelligent learning cannot be promoted [8].

Facial recognition technology refers to determining the identity of the person in the database through the recognition of facial information by intercepting the portrait in the image or video [9]. The wide application value and academic influence of facial recognition have made it develop by leaps and bounds, and it has maintained a high research interest in various fields for many years. As one of the biological features, the human face can intuitively and effectively reflect the differences between individuals and provide effective identification information [10, 11].

At present, facial recognition has received extensive attention from academia and society [12]. There are countless research topics on recognition in various fields in various countries, and it has achieved fairly good results in the well-known face data set [13]. However, most of the traditional facial recognition algorithms are carried out in the case of visible light, but such recognition systems are easily affected by the external environment (light, angle, etc.). When facial recognition algorithms are used in real-world scenarios, their recognition rate will drop significantly. Faced with such a situation, although facial recognition has achieved a relatively high degree of completion technically, theoretically, and practically, there are still many problems to be improved [14]. In order to make facial recognition technology closer to the practical application of life, it is necessary to explore in-depth from multiple directions to find a feasible solution to improve performance [15].

In the new classroom teaching, we should not only pay attention to the teaching content of teachers but also pay attention to the feedback of students. Humanistic psychology emphasizes the importance of students in classroom teaching [16]. “Teaching based on learning” believes that students must be the main body of teachers' teaching quality evaluation, starting from students' classroom learning status, such as students' emotional changes, thinking activity, and participation in classroom learning, as the basis for teaching quality evaluation [17]. Therefore, paying attention to students' classroom learning status is of great significance to strengthen education and teaching and teaching management and improve teaching efficiency.

Through the analysis of teaching videos in educational activities, it is found that the change of students' facial features during the learning process is the most intuitive way to express their psychological state [18]. If the teacher's teaching method is humorous and vivid, then the facial features of the students will show a positive state, so that they will listen to the lectures with passion and earnestness, and the learning efficiency will be greatly improved [19]. But if teachers teach in a monotonous and boring way, students will lose interest in listening to the lectures and show negative facial features [20, 21]. Therefore, it can be seen that the analysis of facial features can effectively understand the students' classroom learning status.

This paper proposes a multiattention method that fuses shallow features with deep features. Shallow features use the relative motion position and texture characteristics of facial key points to briefly describe the feature description of AUs in FACS, while deep features use deep convolutional neural networks to extract high-level semantic features of images and fuse them. In the whole model, we introduce multiple attention mechanisms to improve the recognition effect. This paper demonstrates that by increasing teachers' attention to students and stimulating the positive side of students' academic emotions, students' correct rate of homework completion increases significantly. It shows that the method of this study can provide teachers with students' academic emotions and make adjustments according to the obtained academic emotions to increase incentives and guide students' positive academic emotions, so as to increase the positive side of students' academic emotions. This can be directly related to the improvement of the accuracy of students' question-making and ultimately promote the improvement of students' academic performance.

## 2. Methods

### 2.1. Hadoop Platform Construction

Hadoop is a distributed processing platform deployed on the Linux operating system, which can manage and invoke the resources of multiple hosts at the same time, providing support for large-scale data computing. In this experiment, a Hadoop cluster is built on three hosts, one of which is master and slave nodes, and the other two are slave nodes, which are mainly composed of the following steps.

1. *Basic Installation*. Install the Ubuntu14.04.1 system (64 bits) on each host of the cluster. Since Hadoop2.0 and above are compiled in a 64-bit environment, you need to select the version of the operating system that is also 64 bits.
2. *jdk Installation*. This article selects jdk1.7.09 version to provide the JVM environment required by the Hadoop system and meet the programming needs. After downloading the jdk1.7.09.tar.gz file adapted to the Linux system from the Oracle official website, you use tar –zxvf [file name] command to decompress it to the/Java folder, enter the sudo etc/profile command to open the profile file, and configure the installation path of jdk in it.
3. *Modify the Host Name*. In order to facilitate the later Hadoop environment configuration and distinguish between different nodes, the name of the master node is set to master by modifying the etc/hosts of the node, and the name of the slave node is set to slave1, slave2 in turn, and each node is set at the same time.
4. *SSH Installation*. SSH (Secure Shell) is a security protocol based on the application layer, mainly used for remote login and other network services, which can effectively prevent problems such as information leakage, because the master node needs to coordinate and control the slave nodes when Hadoop is running, so that frequent communication occurs between them. If the password is continuously input during this process, it will cause great trouble. Therefore, it is necessary to configure SSH password-free login for the Hadoop system.
5. *Install Hadoop*. Download the Hadoop-2.5.1 (64 bits) version from the Hadoop official website. After decompression, you first configure the relevant path of jdk to etc/Hadoop/Hadoop-env.sh and then modify the relevant configuration files to configure. The address and port number of the HDFS file system, the number of file backups, and the port number and address of the JobTracker are used to complete the configuration of the Hadoop cluster.

After all the above related content is configured, we first format HDFS with the bin/Hadoop namenode–format command. Then, we use the bin/start-all.sh command to start the Hadoop cluster, and we can use the jps command to check whether all processes of the Hadoop system have been started. According to the configuration of this article, if the Hadoop cluster is successfully started, there will be 5 daemons in the master node.

Considering the actual situation, this paper also sets the master node as the DataNode node. Therefore, a DataNode daemon is also included in the startup process of the master node.

### 2.2. Parallel Processing Optimization of Student Facial Image Data

The default block size in Hadoop 2.0 and above is 128 MB. Generally, files smaller than 128 MB are considered small files. Since the metadata of each file in Hadoop is stored in the memory, storing a large amount of image and small file data requires a lot of memory resources, and it needs to switch between different data nodes when reading files, which seriously affects the cluster. Therefore, the processing speed of massive small files is much lower than the processing speed of large files of the same size. Moreover, in the process of image processing, for the integrity of the image, most of them use one fragment to process one image, and each fragment is completed by a Map task, so processing a large number of small image files will start a large number of maps, resulting in greatly reduced cluster performance. Therefore, when processing image data in the Hadoop platform, we must first solve the memory consumption caused by massive small image files and the impact on cluster processing efficiency. This paper adopts the method of processing small image files into serialized files to optimize the facial image data of students.

#### 2.2.1. Generate SequenceFile

A large number of small image files are packaged into SequenceFile files, which not only does not destroy the structure of image files but also effectively solves the problem of too many Map task startups. It stores multiple image files in the form of binary records.

By specifying the FileSystem object, path object, configuration object, and key and value types, you can get a SequenceFile. Writer instance, then call the append() method to add the <key, value> key-value pair to the end of the file. The value is the content of each picture, so that the purpose of converting multiple small files into SequenceFile files can be realized.

#### 2.2.2. Read SequenceFile

After getting the serialized file, you first create an instance of SequenceFile. The Reader will get the starting position of the file, read the record through sync, read the record in the form of <key, value> key-value pair, and pass it as input to the map function.

You use the SequenceFileInputFormat input format to process the serialized file, call the SequenceFile Record Reader instance, which locates the position of each record according to sync and uses SequenceFile. Reader will read the records into <key, value> key-value pairs in the order in which they were generated. In the experiment of this paper, the key saves the image file name, and the value saves the image content. After being processed by the Map task and the Reduce task, the file is output to the HDFS file system by means of MultipleOutputs.

### 2.3. Design of Parallel Image Processing

A data type is a collection of values and a set of operations defined on this collection. There are 8 data types provided by default in the MapReduce framework. The most commonly used types are Text, IntWritable, NullWritable, and FloatWritable, but there is no definition for images. Therefore, processing images using the Hadoop platform first requires customizing the data types used to store images.

#### 2.3.1. Design of Image Data Type

The Hadoop system is a master-slave architecture model. The master node is responsible for coordinating and unifying the task startup, task execution, and resource recovery of the slave nodes. There are frequent file transfers and information exchanges between nodes. In order to save bandwidth and improve cluster efficiency, Hadoop customized its own serialization method and provided the writable interface. Hadoop requires that all user-defined data types must implement its writable interface. To realize the processing of image files in the Hadoop system, the data type that stores the image must first implement the writable interface. This article customizes the data type raw image for storing images by rewriting the two methods of the writable interface and readFields().

The raw image designed in this paper implements the write() and readFields() methods in the writable interface. At the same time, in order to process images more conveniently, the functions of converting images to Mat types with single channel or three channels and alpha channels and encoding Mat types into image files of different formats are also implemented in combination with Opencv library functions.

#### 2.3.2. Input and Output Format Design

Using the SequenceFileInputFormat input format, the large SequenceFile is cut into multiple slices and handed over to the Map task for processing, and a slice contains multiple records, each record is a picture, the key is the file name of the image, and the value is the image. The FileOutputFormat class is used to describe the format of the output data, and the image data is written to the HDFS file system through the record writer.

The default output file name of Hadoop is in the form of name-r(m)-nnnnn, where name can be customized by the user, r represents the reduce output, m represents the map output, and nnnnn is an integer indicating the block number. To display the image, the output file can be output in the form of file name.jpg. This article rewrites the getDefaultWorkFile() method of the FileOutputFormat class.

### 2.4. Image Feature Description and Extraction

#### 2.4.1. Color Features of Students' Face Images

Color features are based on the analysis of all pixels of the image or each pixel of the target object of interest and can describe the global information of the image. The selection of a color feature must first select the corresponding color space. Among a variety of different color spaces, the HSI color space is widely used because it can more accurately simulate the visual characteristics of the human eye.

The specific values of the pixels on the students' faces are extracted, and the values of some of the pixels are arbitrarily taken from them to observe their distribution, and the data shown in Table 1 is obtained.

In this paper, the low-order moment of Hue (hue) in HSI space is used to describe the color characteristics of students' faces. The expression of the first three-order moment Hue moment is as follows:

(1) $$\begin{array}{c} M_{1}=\frac{1}{N-1}\overset{N-1}{\underset{i=0}{\sum }}H\left(p_{i}\right), \end{array}$$

(2) $$\begin{array}{c} M_{2}={\left\{\frac{1}{N-1}\overset{N-1}{\underset{i=0}{\sum }}{\left[M_{1}-H\left(p_{i}\right)\right]}^{2}\right\}}^{1/2}, \end{array}$$

(3) $$\begin{array}{c} M_{3}={\left\{\frac{1}{N-1}\overset{N-1}{\underset{i=0}{\sum }}{\left[M_{1}-H\left(p_{i}\right)\right]}^{3}\right\}}^{1/3}. \end{array}$$

In the above formula, *N* represents the number of pixels in the segmented student face image, and *H*(*pi*) represents the Hue component value of the *i* student face pixels in the HSI space in the student face image segmentation region *p*.

#### 2.4.2. Texture Features of Students' Face Images

Texture is a feature that reflects the periodic regularity or slowly changing properties of the surface of an object. Unlike the color feature that describes an image based on a single pixel, it describes the image through the distribution of pixels. It has scale and rotation invariance and is resistant to noise. It also has strong resistance, and the distribution, roughness, uniformity, etc., of the image surface material can be reflected by texture features. When the color of students' faces and distractors are similar, texture features can be used to distinguish their spatial distribution and structural information, so as to further identify students' faces.

#### 2.4.3. Sift Features of Student Face Images

Different from color features and texture features, the Sift (Scale Invariant Feature Transform) feature is a feature that remains invariant to scale scaling, rotation, and brightness and is also good for viewing angle changes, noise, occlusion, and other interference factors.

To find the feature points on the image, first, convert the image from grayscale space to Gaussian difference scale space. The conversion formula is as follows:

(4) $$\begin{array}{c} D\left(x^{\prime },y;\sigma \right)=I\left(x,y\right)*\left|G\left(x,y;\sigma \right)-G\left(x,-y;k\sigma \right)\right|. \end{array}$$

Among them, *D* represents the Gaussian difference function, *x*′ represents the position of the extreme point, and the point *D*(*x*′) lower than the threshold is eliminated by setting the threshold. (*x*′, *y*) represents the position of the pixel, and *σ* and ∗ represent the spatial scale factor and convolution operation, respectively. In the Gaussian difference scale space, a pixel is compared with 26 points in the 3 × 3 domain of its upper and lower adjacent scales. If this point is the maximum point or the minimum point, then it is considered as an extreme point.

The extreme point detected in the first step is the extreme point in the discrete space, and the low contrast and unstable edge points need to be eliminated by the function to further enhance the antinoise ability.

(5) $$\begin{array}{c} m\left(x,y\right)={\left\{{\left[\left(x,y-1\right)-L\left(x-1,y-1\right)\right]}^{2}+{\left[L\left(x,y+1\right)-L\left(x-1,y-1\right)\right]}^{2}\right\}}^{1/2}, \end{array}$$

(6) $$\begin{array}{c} \theta \left(x,y\right)=\frac{\left[L\left(x-1,y-1\right)-L\left(x+1,y\right)\right]}{\left[L\left(x-1,y\right)-L\left(x+1,y+1\right)\right]}. \end{array}$$

There may be more than one direction for the extreme point obtained by positioning. In order to ensure that the descriptor has rotation invariance, the stable direction of the extreme point is obtained by calculating the gradient of the image. After the gradient calculation is completed, the gradient and direction of the pixels in the point field are calculated and represented by a histogram, and the peak direction of the histogram is marked as the direction of the extreme point.

Through the above 3 steps, the position, direction, and scale information of each extreme point are obtained. At this time, the 16∗16 field around the extreme point is divided into 4∗4 submodules, and the gradients in the 8 directions of each submodule are calculated, respectively.

### 2.5. Facial Expression Recognition with Multiattention Fusion Network

Shallow features can leverage people's prior knowledge about facial expression recognition tasks, while deep features can express high-level semantic features of images. In order to take full advantage of the advantages of these two features, it is necessary to combine these two features to realize a dynamic sequential facial expression recognition system.

Therefore, this paper proposes a dynamic sequential facial expression recognition system that combines shallow and deep features with multiple attention mechanisms. The shallow attention model (ASModel) extracts shallow features of AU-based images by describing the relative positions of facial landmarks and the texture features of local regions. At the same time, using the advantages of CNNs in expressing high-level features of images, a deep attention model (ADModel) is designed to extract the deep features of sequence images by improving the ALexNet structure.

The multiattention fusion model (MSDModel) is combined with the shallow attention model and the deep attention model to realize the dynamic sequence facial expression recognition. To strengthen the connection between image sequence features and improve the effectiveness of the model, three attention mechanisms are introduced: self-attention (SA), weight-attention (WA), and convolue-attention (CA). SA is the input data through attention matrix, WA uses weighted matrix to achieve the alignment of feature sequences, and CA is introduced through convolution operation, so that you can process the sequence image data of CNN. A feature vector *X* can be extracted from each face image. Then, a dynamic sequence of images of length *L* can be composed of a feature matrix, denoted as [*X*_1_, *X*_2_, ⋯,*X*_*t*_, ⋯,*X*_*L*_]^*T*^, where *t* is the *t*-th image. In order to understand the influence of other frames on the original feature vector of the current frame, a self-attention mechanism (SA) is introduced. SA achieves the degree of influence between shallow features of different frames by introducing a self-attention matrix (SAMat). Values on the diagonal of this matrix are initialized to 1, and other values are initialized to 0. FC represents a fully connected layer, and C is the category of the dataset's expression category, and *O*_1_ is the output of the shallow model. The calculation method of SA can be expressed as follows:

(7) $$\begin{array}{c} X_{t}^{\prime }=\overset{m-1}{\underset{i=0}{\prod }}\left(x_{t}*x_{t+1}*{\text{SAMat}}_{ti}\right). \end{array}$$

In the processing of image *t*, the forward LSTM can only combine the image change information from 1 to *t* − 1. However, when dealing with image *t*, it is best to also consider the expression change relationship of the image from *t* + 1 to *L*. Therefore, a bidirectional LSTM (BiLSTM) is used to process the SA-processed feature matrix.

Although CNNs have achieved state-of-the-art results in various vision tasks, they generally work on 2D planar images. The AlexNet structure is improved to handle 3D spatiotemporal image sequences. Conv is a convolutional layer, pool is a pooling layer, FC is a fully connected layer, and C is an emotion type. *O*_2_ is the output of the deep model. Here we have two areas for improvement. First, the first layer of convolution and pooling is extended to sequential mode, i.e., the same convolution and pooling operations are performed on each image with shared parameters. Then, the convolution operation is performed through CA and a 1-by-1 convolution kernel, and the above calculation results are accumulated to eliminate the time dimension. CA can be calculated using the following formula:

(8) $$\begin{array}{c} \text{CA}\left({\text{CP}}_{t}{\text{CA}}_{t}\right)=\frac{1}{L-1}\overset{L-1}{\underset{t=0}{\prod }}\left({\text{CP}}_{t}⊗{\text{CA}}_{t}⊗{\text{CP}}_{t+1}⊗{\text{CA}}_{t+1}\right). \end{array}$$

Among them, ⊗ represents the convolution operation, CA_*t*_ is the 1-by-1 convolution kernel, CP_*t*_ is the output of the previous layer, and *L* is the length of the sample image sequence.

Figure 1 shows the data flow for the fusion of the two models, where *WA* is calculated as follows:

(9) $$\begin{array}{c} F\left(O_{1},O_{2};\;W_{1},W_{2}\right)=\frac{\left|W_{1}^{T}O_{1}+W_{2}^{T}O_{2}\right|}{2}. \end{array}$$

When training ASModel, the input is a shallow feature matrix, and the output is *O*_1_; when training ADModel, the input is a sequence of facial expression images, and the output is *O*_2_. When training MSDModel, the input is a shallow feature matrix and a sequence of facial expression images, and the output is *F*.

## 3. Results

### 3.1. Comparison of Running Time

In order to verify the time performance of the parallelized algorithm, this paper uses 500-3000 image datasets to test the running time of the feature extraction algorithm under different node conditions. Taking the extraction of Sift features of images as the experimental background, the time-consuming situation of extracting Sift features of different image datasets under different nodes is obtained. The results are shown in Figure 2.

When the number of images is small, the time-consuming difference of image feature extraction under different nodes is not obvious. This is because the multinode cluster architecture increases the communication overhead between node computers, which will lead to the processing of small-scale image datasets. It can sometimes take longer to run than a single-node computer can handle. With the sharp increase in the number of images, the advantages of the Hadoop cluster computer system with multinode architecture are gradually reflected, although the running time of the algorithm will fluctuate with the increase of the number of images in different nodes. However, it can be seen that the running time of the 2-node computer processing is the largest, while the increasing trend of the running time of the computer system of the cluster architecture is relatively gentle. The higher the number of node computers, the lower the running time, which fully proves the superiority of the Hadoop cluster architecture in processing massive image data.

### 3.2. Comparison of Speedup Ratio

Speedup ratio refers to the ratio of the running time of the same task in a single-node environment to that in a multinode environment and is an important indicator to measure the efficiency of parallel algorithms under the Hadoop platform. In order to verify the performance of the proposed algorithm under the Hadoop platform, this paper selects 500-3000 students' facial image data from the constructed student face image database to test the speedup ratio on different nodes. The results are shown in Figure 3.

Due to communication overhead and load balancing, the speedup ratio cannot actually increase linearly. Under the number of 500~3000 images, the acceleration ratio of the system increases with the increase of node computers, and the growth rate is larger, which further fully shows that the Hadoop cluster can better reflect its superiority in processing large-scale data sets. Furthermore, the system speedup fluctuates as the number of images increases.

### 3.3. Results Analysis of Students' Facial Expression Recognition and Academic Emotions

In each class, data is set to be intercepted from the video stream every 4.9 seconds. At the end of a class, 550 valid data will be obtained, 3,300 valid data will be obtained every week, and 26,400 valid data will be obtained at the end of the practice. Identifiable data is in units of each lesson hour.

It can be seen from Figure 4 that the recognition rate of practice data is as low as 80% and as high as 92%. From this, it can be concluded that the data recognition rate collected in the actual classroom is relatively high and meets the expected requirements of practice. In addition, the recognition rate of the multiattention fusion network proposed in this paper is higher than that of the deep attention network, and the recognition rate of the deep attention network is higher than that of the shallow attention network.

The result analysis of academic emotion in the classroom mainly quantifies the academic emotion in the classroom. The quantified academic emotion can be analyzed in many aspects. In this study, we focus on the change of academic emotion.  Figure 5 shows the change of academic mood in 45 minutes.

At the beginning of the class, the number of students in positive emotions is not high, indicating that students have not transitioned from the state of rest between classes to the state of class in class. The number of students who were in a positive mood before the end of get out of class fell back to a state similar to that at the beginning of the class. This time period is the time for summarizing knowledge points and leaving homework.

With the learning of new knowledge points in the middle of the classroom, the number of students in positive emotions generally increases, but the number of students fluctuates, which shows that students' emotions fluctuate and change when they encounter difficult problems during the explanation of new knowledge points. Related research in educational psychology shows that the attention span of teenagers in classroom learning is about 25 minutes [12]. When students are in the time of attention, the positive academic mood is also relatively increased; when the students are in the time of distraction, the positive academic mood is also relatively reduced.

From an overall point of view, the changes of students' academic emotions in normal classroom teaching activities in natural state will be less changes at the beginning of the class, mostly calm academic emotions, and gradually change with the increase of teaching time. Teachers play a significant role in stimulating and transforming students' academic emotions in the classroom.

### 3.4. The Correlation between Academic Mood, Academic Performance, and Teaching Effect

In practice data statistics, the focus is on the statistics of students' academic mood and learning situation, as detailed in Table 2. It can be seen from Table 2 that the academic sentiment has been increasing over time, with the highest value in the seventh week, and the review of the final exam is relatively tight in the seventh week. The lowest value appeared in the first week. The learning situation of the students in this week was adjusted by the teacher at the beginning to stimulate the positive academic mood of the students. It can be seen that the teacher has a significant effect on the positive academic mood of the students, and it increases significantly over time. From the completion of the homework, the homework can be completed when the teacher pays attention, but the increase in the accuracy of the homework is not particularly obvious, although it has increased.

## 4. Discussion

### 4.1. Recognition of Facial Expressions with Different Emotional Types

When recognizing emotional faces with complete facial feature information or emotional faces with incomplete facial feature information, happy emotion has the advantages of high accuracy rate and short response time compared with the other six emotions, and its recognition accuracy rate is significantly higher than that of the other six emotions [22, 23]. The other 6 emotions, followed by neutral emotions such as calm, while negative emotions such as sadness, anger, disgust, and fear, are more difficult to identify [15, 24]. Among them, fear and disgust are the most difficult emotions to identify. Their accuracy is low and their response time is significantly longer than that of other emotions [25]. This is basically consistent with previous studies, especially a large number of studies have shown that positive emotions such as happiness are better than other negative emotions. The recognition of different emotional types is different, which can be verified from the development of primary school students in emotional recognition [26–28].

Relevant scholars used the verbal naming task to ask pupils to name expressions and select the corresponding expressions from four expressions [29, 30]. The results show that the ability of pupils to name and identify happy emotions is better than the ability to identify negative emotions. Among the negative emotion abilities of naming and recognizing, the fear emotion is the most difficult for elementary school students to recognize [31–33]. The same results were obtained in a study of Asian, Mexican, and Caucasian American elementary school students. Facial expressions are innate, such as babies smiling and crying from birth, and the ease of recognizing happy emotions is a result of human evolution. Happy emotional facial expression is a face that can be seen almost every day in daily life, and it has the highest frequency of use among all emotional faces. Many researchers believe that it is this difference in frequency that accounts for the differences in facial expression recognition performance between different emotion types [21, 27, 30].

Positive emotional facial expressions are more standardized and have simpler visual features than negative emotional facial expressions. For example, the corners of the mouth that are raised upwards can be quickly associated with happy emotions. When the mouth is wide open and the eyes are shining, the expression of surprise can be immediately associated with it, while the negative emotions are more diverse and complicated, and it is difficult to extract enough from a single feature.

### 4.2. Features of Recognition of Emotional Facial Expressions with Different Difficulties

When facial information is presented incompletely, emotional facial expression recognition is affected by the amount of facial feature information presented [34, 35]. The more facial information is presented, the higher the recognition accuracy is, and the less the facial information is presented, the lower the recognition accuracy is. The amount of information presented on the face has a greater impact on the recognition of these two emotions [36].

It is difficult to identify students' calmness and anger by relying on one feature part information alone, but if one more feature part information is presented, that is, two feature part information can be better recognized and the recognition performance when presenting a complete face is not much different [37, 38]. The angry expressions of primary school students can achieve the same effect as the information of three characteristic parts when they present the information of two characteristic parts, while the angry expressions of college students are different.

The recognition accuracy rate is much higher when three feature part information is presented than when two feature part information is presented. This may be due to the fact that the information of a single feature part of the student's face has a large correlation with positive emotions and a small correlation with negative emotions. In other words, a single feature part of the face can well reflect positive emotions, and the combination of multiple feature part information can better reflect negative emotions.

### 4.3. Recognition of Emotional Facial Expressions Presenting Different Facial Part Features

The recognition of sadness and fear is more dependent on the information provided by the eyes, the recognition of surprise and calm emotions is more dependent on the information provided by the mouth, and the recognition of happiness, anger, and disgust is more dependent on the eyes and mouth [39–41]. The degree of dependence on the provided information is indistinguishable, among which the recognition of happy and angry emotions relies more on eye information, and the recognition of disgust emotions relies more on mouth information [42, 43].

This also differs in recognizing the emotional facial expressions of college students and elementary school students. When recognizing the emotional facial expressions of elementary school students, the recognition of sadness and anger depends more on the information provided by the eyes; the recognition of calm and disgust depends more on the information provided by the mouth, while the eyes and mouth are more sensitive to happiness [44, 45]. When recognizing the emotional facial expressions of college students, the recognition of sadness and fear is more dependent on the information provided by the eyes; the recognition of surprise, calm, and anger is more dependent on the information provided by the mouth, while happiness and disgust are more dependent on the information provided by the mouth [46–48]. The recognition depends on the eye and mouth information to the same extent. It can be seen from this that the facial feature information relied on is different when recognizing the different emotional facial expressions of college students and primary school students [49].

## 5. Conclusion

Experiments show that the proposed feature extraction algorithm based on Hadoop platform can effectively extract the features of large-scale massive images, and it takes less time to run, and the algorithm acceleration is ideal. The built Hadoop cluster can make full use of the resources of each node computer. Compared with a single-node computer, it fully reflects the powerful computing power of the distributed parallel processing of the Hadoop cluster. After the practice of this research and the analysis of the results of the practice, the obtained practice results show that the practice has realized the mining and analysis of academic emotions based on the recognition of students' facial expressions. In order to summarize the research and draw the conclusion of the research and fully demonstrate and analyze the correlation, a traditional scale questionnaire was made. The results of the analysis found that the results of the study were consistent with the actual situation, demonstrating the validity of the study. To verify that this study can support and serve as a basis for follow-up research, a study on the impact of academic emotions on academic performance was conducted. The results suggest that the study can provide teachers with feedback on students' academic mood. After receiving the results of students' academic emotions, teachers can effectively promote students' academic performance after adjustment. The practical results of the research on the impact of academic emotions on academic performance demonstrate that this research can be used as the basis for follow-up research and can provide support for follow-up research.

## Figures and Tables

**Figure 1:** Fusion model of shallow and deep networks.

**Figure 2:** Run time comparison.

**Figure 3:** Comparison of speedup ratios.

**Figure 4:** Practical data identifiability rate.

**Figure 5:** Academic mood changes in 45 minutes.

**Table 1:** Values of some students' face pixels in HSI space.

Weight	H	S	I
Face pixel 1	37	112	192
Face pixel 2	38	104	189
Face pixel 3	41	108	191
Face pixel 4	39	107	187
Face pixel 5	45	112	193
Face pixel 6	42	110	188

**Table 2:** Statistical table of academic mood and learning situation.

Week number	1	2	3	4	5	6	7	8
Time (min)	51	103	97	156	142	131	173	138
Degree of completion	0.98	0.99	1	0.99	1	1	0.99	1
Accuracy	0.71	0.75	0.79	0.74	0.76	0.87	0.89	0.86

## Data Availability

The data used to support the findings of this study are available from the corresponding author upon request.
